The article "The scalability of common paradigms for assessment of cognitive function: A functional transcranial Doppler study" was published in 2022. Journal: PLoS One.

# The scalability of common paradigms for assessment of cognitive function: A functional transcranial Doppler study

**DOI:** 10.1371/journal.pone.0266048

**Published:** 2022-03-28

**Authors:** Kannakorn Intharakham, Ronney B. Panerai, Thompson G. Robinson

**Affiliations:** 1 Department of Cardiovascular Sciences, University of Leicester, Leicester, United Kingdom; 2 NIHR Leicester Biomedical Research Centre, British Heart Foundation Cardiovascular Research Centre, Glenfield Hospital, Leicester, United Kingdom; University of Caytania, ITALY

## Abstract

Cognitive paradigms induce changes in cerebral blood flow (CBF) associated with increased metabolic demand, namely neurovascular coupling (NVC). We tested the hypothesis that the effect of complexity and duration of cognitive paradigms will either enhance or inhibit the NVC response. Bilateral CBF velocity (CBFV) in the middle cerebral arteries (MCAs) via transcranial Doppler ultrasound (TCD), blood pressure (BP), electrocardiogram (ECG) and end-tidal CO_2_ (EtCO_2_) of 16 healthy participants (aged 21–71 years) were simultaneously recorded at rest and during randomized paradigms of different complexities (naming words beginning with P-,R-,V- words and serial subtractions of 100–2,100–7,1000–17), and durations (5s, 30s and 60s). CBFV responses were population mean normalized from a 30-s baseline period prior to task initiation. A significant increase in bilateral CBFV response was observed at the start of all paradigms and provided a similar pattern in most responses, irrespective of complexity or duration. Although significant inter-hemispherical differences were found during performance of R-word and all serial subtraction paradigms, no lateralisation was observed in more complex naming word tasks. Also, the effect of duration was manifested at late stages of 100–7, but not for other paradigms. CBFV responses could not distinguish different levels of complexity or duration with a single presentation of the cognitive paradigm. Further studies of the ordinal scalability of the NVC response are needed with more advanced modelling techniques, or different types of neural stimulation.

## Introduction

Neurovascular coupling (NVC) describes the mechanism of cerebral blood flow (CBF) regulation through changes in arteriolar and capillary diameter to match increasing metabolic demand during neural activation [1, 2]. Action potentials, resulting from neural stimulation, release neurotransmitters to the neurovascular unit (neurons, astrocytes, pericytes, endothelial cells and extracellular matrix components), where neuronal mediators, such as K^+^, NO and adenosine, control vascular smooth muscle contraction or relaxation [3–5]. CBF changes in response to cognitive task activations can be studied with a number of non-invasive methods, including magnetic resonance imaging (MRI) [6], positron emission tomography (PET) [7], single-photon emission computed tomography (SPECT) [8], near infrared spectroscopy (NIRS) [9], laser Doppler flowmetry [10] and transcranial Doppler ultrasound (TCD) [11]. MRI, PET and SPECT may cause patient discomfort, and are not suitable for screening and follow-up studies. However, TCD can measure CBF velocity (CBFV) at rest, or during cognitive tasks, usually referred to as functional TCD (fTCD) [12]. fTCD has multiple advantages in terms of low-cost, high temporal resolution, portability to the bedside and non-harmful repetitive studies. Therefore, current TCD applications have been adopted to study a wide range of conditions such as sickle cell disease [13], ischaemic [14] or haemorrhagic [15] stroke, brain stem death [16], intraoperative monitoring [17], cerebral microembolism in right-to-left cardiac shunt [18], and cognitive impairment [19], including cerebral pressure autoregulation [20] and neuroactivation [21]. The quantification of the NVC response has been assessed by CBFV changes (ΔCBFV), induced by neural stimulation [12, 22–25]. Moreover, fTCD has been extensively used for assessing NVC in the lateralization of functional brain regions with a range of tasks, such as cognitive [23, 26–28], visual [11, 29, 30] and sensorimotor [24, 31, 32] paradigms.

The article "The scalability of common paradigms for assessment of cognitive function: A functional transcranial Doppler study" was published in 2022. Journal: PLoS One.

In addition to detecting differences in lateralisation, a diagnostic tool to assess cognitive function needs to satisfy the condition of *scalability*, that is, to demonstrate the sensitivity to reflect differences in cognitive load, or its complexity. In the case of fTCD, this has been shown to be the case with visual stimulation [30, 33], with changes in ΔCBFV detected in the posterior cerebral artery (PCA). With cognitive paradigms though, evidence of scalability is limited, and far from generalizable. In a few studies, fTCD has shown sensitivity to detect differences in difficulty and cognitive load, with the use of n-back paradigms [28, 34, 35]. The n-back paradigm stimulates specific aspects of cognition, involving attention and short-memory [36], but does not involve other aspects of cognitive function, such as language, fluency and visuospatial domains, which are part of a more comprehensive assessment of cognitive function [37–39]. Previous studies have shown that fTCD can detect the NVC response to all five main cognitive domains of the Addenbrooke’s Cognitive Examination (ACE-III) battery of tests, an important step to demonstrate the way fTCD might contribute to improving the diagnostic accuracy of routine cognitive assessment [26, 40, 41]. Given that the ACE-III battery involves 20 different tasks, assessing the scalability of each of these paradigms is beyond the capacity of a single study. As a first step, we have chosen to study the scalability of naming words (NW) and serial subtraction (SS) as these tasks have been shown to induce consistent CBFV responses [26, 41] and good reproducibility [40]. The relevance of NW and SS is that they are part, not only of the ACE-III, but also of other current methods of cognitive assessment such as the Mini Mental State Examination (MMSE) and Montreal Cognitive Assessment (MoCA) [37–39].

The article "The scalability of common paradigms for assessment of cognitive function: A functional transcranial Doppler study" was published in 2022. Journal: PLoS One.

In summary, we tested the hypotheses that the complexity and duration of stimulation of NW and SS tasks can: 1) induce either larger or smaller magnitude of NVC response, and 2) lead to inter-hemispherical differences that could be the consequence of either enhanced or inhibitory mechanisms.

## Materials and methods

### Subjects and measurements

Sixteen healthy participants (eight women) without history of cardiovascular, neurological, or respiratory conditions, including metabolic abnormalities, inflammatory abnormalities, and severe somatic (e.g., cancer) or psychiatric (e.g., psychotic or bipolar), were recruited from the University of Leicester as students or staff. The Research Ethics committee approved the study (ref: 19452-rp9-ls:cardiovascularsciences), and fully informed, written consent was signed by each participant. Only adults 18 years old or older, with good insonation of bilateral temporal windows were suitable for study inclusion. The Edinburgh inventory was used for assessment of handedness [42].

All participants abstained from caffeine, alcohol, vigorous exercise, heavy meal, and smoking for at least 4 hrs before attending a temperature (22–24°C) and light controlled laboratory. All measurements were undertaken with participants in the seated position. To avoid any artefacts due to movement, participants were asked to sit comfortably and avoid any movement, and all signals were checked prior to recording. The 2MHz TCD probes (Viasys Companion III device) were securely placed over the temporal windows using a head frame, and bilateral CBFV was monitored continuously in the middle cerebral artery (MCA) with the depth of insonation at 45–55 mm. Arterial volume clamping of the left middle finger digital artery was used for continuous beat-to-beat BP measurement (Finometer, Finapres Medical Systems; Amsterdam, the Netherlands), and automated brachial BP was also intermittently recorded in the right arm to calibrate the Finometer before each recording, using a validated OMRON (UA767) device. Continuous measurements were recorded for heart rate (HR), with a three-lead electrocardiography (ECG), respiratory rate and end-tidal CO_2_ (EtCO_2_), using small nasal cannula (Salter Labs, ref 4000) with a capnograph (Capnocheck Plus).

The article "The scalability of common paradigms for assessment of cognitive function: A functional transcranial Doppler study" was published in 2022. Journal: PLoS One.

### Paradigms of different complexity and duration

Prior to the tests, the paradigms were described in detail, and participants were encouraged to provide their best mental effort when providing their answers in a low voice. Each paradigm was recorded during 60s with subjects asked to keep an ‘empty mind’, Tasks were given verbally to participants during recording before task initiation. Thereafter, paradigms were performed over one of three different periods of duration stimulation, with a 60s recovery phase. Naming words (e.g. P-words) and serial number subtraction (subtract sequentially 7 from 100) paradigms have been applied routinely for diagnosing mild cognitive impairment (MCI) and dementia, and have been increasingly adopted as equivalent cognitive paradigms for assessment of NVC and also functional cerebral lateralization [26, 41]. Hence, both types of paradigms were modified to determine the effect of complexity and duration in this study. For modulating intensity of neuronal activations, naming words (NW) beginning with P-, R- and V- were adopted to represent increasing levels of difficulty corresponding to easy, moderate and hard, respectively [43]. Also, three levels of difficulty in sequential subtractions (SS) were created with SS of (100–2), (100–7) and (1000–17), respectively (Fig 1).

**Fig 1:** Protocol and experimental setup. Changes in cerebral haemodynamics were recording with transcranial Doppler (TCD) insonated bilateral middle cerebral arteries (MCAs) during cognitive stimulation. Blood pressure (BP), Heart rate (HR) and End-tidal CO_2_ (EtCO_2_) were simultaneously recorded.

Subjects rested for 15 min and a resting baseline recording was performed for 5 min (Fig 1). Two separate continuous recordings of cognitive paradigms were then obtained for duration and complexity data. R-words and subtraction (100–7) were used as a reference for representing word-naming (NW_REF_) and serial subtraction (SS_REF_), respectively. Paradigms of different complexity were randomized and presented during 60s. For changing the duration of presentation, the NW_REF_ and SS_REF_ paradigms were also randomised and then interrupted after 5, 30 or 60s, without participants’ prior knowledge. The 60 s has been the traditional duration of NW and SS tasks [26, 41], but a plateau is usually observed from 30 s onwards and using 5 s would only detect the potential effects of central command, before the metabolic deficit starts to act as a feedback error to correct the need for additional O_2_ supply. The beginning and end of stimulation were marked with an on/off electrical switch to identify the duration of the paradigm and allow synchronization for coherent averaging of CBFV responses. All physiological signals were sampled at 500 Hz and recorded in the PHYSIDAS data acquisition system (Department of Medical Physics, University Hospitals of Leicester NHS Trust, Leicester, UK) for offline analysis.

The article "The scalability of common paradigms for assessment of cognitive function: A functional transcranial Doppler study" was published in 2022. Journal: PLoS One.

### Data analysis

BP was calibrated at the beginning of each recording, and all signals were visually inspected to identify artefacts, with narrow (<0.1s) spikes, which were linearly interpolated. Bilateral CBFV signals were passed through a median filter with a window width of five samples to remove random noise. All signals were low-pass filtered by a zero-phase Butterworth filter with a cut-off frequency of 20 Hz. RR interval was automatically marked from the ECG, and HR was continuously plotted against time and manually corrected under visual inspection in case of missed markings. Mean values of CBFV and BP were calculated for each cardiac cycle. Linear interpolation was applied to obtain estimates of EtCO_2_ synchronized to the end of each cardiac cycle. Beat-to-beat data were spline-interpolated with a third order polynomial and resampled at 5 Hz to obtain signals with a uniform time base.

Each variable was synchronized by the start of each paradigm, to obtain the coherent average of CBFV for each subject. Bilateral CBFV were expressed in percent (%) by normalization by the 30s of baseline before the paradigm activation. The synchronization placed the beginning of each paradigm at 60s, within a window of 180s duration. Only bilateral CBFV signals were averaged for 10s during five time segments, with the beginning of stimulation starting at 60s: baseline (T1) at 40-50s, (T2) at 60-70s, (T3) at 110-120s, (T4) at 120-130s, and (T5) at 160-170s. Therefore, T1 represents baseline values before stimulation, T2 the immediate response to stimulation, T3 the sustained response, T4 near the end of the response (for 60 s duration of stimulation) and T5 during recovery. All timepoints were fixed for all paradigms, independently of the duration of presentation.

### Statistical analysis

All data were tested for normality using Shapiro-Wilk test. Continuous data with a Gaussian distribution are presented as mean (SD). Outliers of parameters were determined by using the boxplot with interquartile limits between 25^th^ and 75^th^ percentile (interquartile range, IQR) for indicating extreme values beyond 1.5 times (above or below) of the IQR as outliers which were modified by replacing the second smallest or largest values in observations to the threshold boundaries as recommended in Winsorization [44]. Paired t-test (parametric data) or Wilcoxon test (nonparametric data) were used to detect differences in hemispherical comparisons of CBFV response to each paradigm. Two-way ANOVA was adopted to test for differences between time segments and paradigms for interaction in each bilateral hemisphere. Post hoc analysis with Tukey‘s was applied for multiple comparisons. Analyses were conducted using SPSS version 25 for Windows or Graphpad Prism version 9.2 for Windows. Statistical significance was adopted at a value of p < 0.05.

The article "The scalability of common paradigms for assessment of cognitive function: A functional transcranial Doppler study" was published in 2022. Journal: PLoS One.

## Results

Sixteen healthy participants (eight women) were recruited (mean age 31.6 years, [range 21–71 years] and mean BMI 22.6 ± 3.0 kg/cm^2^), and completed all the NW and SS paradigms of variable duration and complexity. A majority of participants (n = 14) were right-handed and two subjects were ambidextrous, following assessment with the Edinburgh handedness inventory. Half of all participants had Asian background, six were Caucasian, and two subjects had Caribbean and African ancestry, respectively. Eight people abstained from alcohol and two subjects were current smokers. Absolute mean (SD) values of baseline CBFV did not show a significant difference between right hemisphere (RH) and left hemisphere (LH) at 66.8 (11.4) and 64.8 (11.4) cm/s, respectively. Baseline values for mean BP, HR and EtCO_2_ were 89.7 (9.4) mmHg, 70.8 (8.1) bpm and 38.5 (3.1) mmHg, respectively.

### Temporal CBFV responses during cognitive paradigms

The overall paradigm-synchronized patterns of bilateral cerebral haemodynamic coherent averages for the whole population with increasing complexity of NW (Fig 2A–2C) and SS (Fig 2D–2F) showed considerable similarity. A rapid increase in bilateral CBFV was observed at the start of stimulation (grey bar), with the largest peak around T2 and reducing rapidly towards baseline values before T3, around 25s after stimulation. There was a further small rise in CBFV around T3, except for SS (100–2), and a steady return to baseline after the paradigm was completed at approximately 20s. The 2-way ANOVA confirmed a highly significant effect of time for NW and SS (Fig 2 and Table 1, p < 0.001).

**Fig 2:** Average population responses (n = 16) in the right (continuous line) and left (dashed line) hemispheres for the complexity of NW (A, B, C) and SS (D, E, F) paradigms of CBFV, respectively. Error bar represents the largest ±SD at the point of occurrence. Changes are shown before, during (grey bar) and after 60s of P-word (A), R-word (B), V-word (C), 100–2 (D), 100–7 (E) and 1000–17 (F). Responses were synchronized by the beginning of stimulation, set at 60s. For statistical analyses, shorter segments (T1-T5) were averaged from 40-50s (T1), 60-70s (T2), 110-120s (T3), 120-130s (T4) and 160-170s (T5), respectively.

The article "The scalability of common paradigms for assessment of cognitive function: A functional transcranial Doppler study" was published in 2022. Journal: PLoS One.

**Table 1:** Mean (SD) values of bilateral cerebral hemodynamic changes at each timepoint for increasing complexity of NW and SS paradigms.

**CBFV**_**RH**_ **(%)**						**Variation (p-value)**		
**NW**	**T1**	**T2**	**T3**	**T4**	**T5**	Interaction	Timepoints	Paradigms
P-word	-0.6(1.4)	7.5(5.8)^a^	0.9(7.7)^b^*	2.8(8.4)^b^	-0.9(5.2)^b^^c^	0.58	**<0.0001**	0.0604
R-word	-1.3(1.7)	6.1(3.7)^a^	-2.2(5.9)^b^	-0.6(6.3)^b^	-2.9(4.3)^b^			
V-word	-0.3(1.1)	8.8(5.3)^a^	1.3(8.0)^b^	1.1(6.4)^b^	-1.8(3.9)^b^			
**SS**	**T1**	**T2**	**T3**	**T4**	**T5**	Interaction	Timepoints	Paradigms
100–2	-0.6(1.2)	6.9(4.0)^a^	3.0(7.4)	2.6(7.5)*	-0.3(4.6)^b^	0.52	**<0.0001**	0.85
100–7	-1.0(1.6)	4.1(4.9)^a^	3.8(6.9)^a^	3.8(9.1)*	-0.4(8.1)^b^			
1000–17	-0.9(1.1)	6.7(5.7)^a^	3.0(8.8)	3.3(9.4)	2.1(3.1)^b^*			
**CBFV**_**LH**_ **(%)**						**Variation (p-value)**		
**NW**	**T1**	**T2**	**T3**	**T4**	**T5**	Interaction	Timepoints	Paradigms
P-word	-0.8(1.1)	7.2(6.0)^a^	3.1(8.6)^a^^b^	4.0(6.7)^a^	0.4(5.6)^b^^c^	0.13	**<0.0001**	0.12
R-word	-1.2(1.5)	6.7(2.9)^a^	0.8(7.9)^b^	0.1(6.1)^b^	-3.2(6.1)^b^			
V-word	-0.5(1.1)	8.5(3.4)^a^	1.8(6.5)^b^	0.5(5.6)^b^	-2.6(2.9)^b^			
**SS**	**T1**	**T2**	**T3**	**T4**	**T5**	Interaction	Timepoints	Paradigms
100–2	0.4(1.3)	6.1(2.7)^a^	1.3(6.9)^b^	0.6(7.4)^b^	-0.2(4.9)^b^	0.56	**<0.0001**	0.90
100–7	-1.1(1.3)	4.2(3.5)^a^	3.1(6.9)^a^	2.0(8.6)	-1.1(6.8)^b^^c^			
1000–17	-0.3(1.1)	6.0(4.8)^a^	2.3(8.0)	2.8(8.1)	-0.8(5.2)^b^			

CBFV was bilaterally normalized at baseline values. Sample size = 16, T1-T5 represents each extracted timepoint for statistical analyses. Interaction showed p-value of paradigm x timepoint effect by two-way repeated measures ANOVA followed by post-hoc analysis with Tukey’s multiple comparison. CBFV; cerebral blood flow velocity, RH; right hemisphere, LH; left hemisphere. NW; naming word, SS; sequential subtraction

^a^ p < 0.05 for difference compared with baseline (after Tukey correction)

^b^ p < 0.05 for difference compared other timepoints with T2 (after Tukey correction)

^c^ p < 0.05 for difference compared with previous time segment (after Tukey correction)

* p < 0.05 for difference between interhemispheric comparisons

Changes in paradigm duration, also led to similar patterns of the CBFV bilateral coherent averages, for both the NW_REF_ (R-word) (Fig 3A–3C) and SS_REF_ (100–7) tasks (Fig 3D–3F). A steep increase to the highest peak at T2 for all durations was observed bilaterally. Thereafter, there was a reduction to baseline, though a rebound increase in bilateral CBFV to a second peak at T3 was seen for the 60s duration paradigm. The 2-way ANOVA corroborated the change in bilateral CBFV response to different duration stimulations, with a highly significant effect of time for NW_REF_ and SS_REF_ (Table 2, p < 0.001).

The article "The scalability of common paradigms for assessment of cognitive function: A functional transcranial Doppler study" was published in 2022. Journal: PLoS One.

**Fig 3:** Average population responses (n = 16) in the right (continuous line) and left (dashed line) hemispheres for the duration of NW_REF_; R-word (A, B, C) and SS_REF_; 100–7 (D, E, F) paradigms of CBFV, respectively. Error bar represents the largest ±SD at the point of occurrence. Changes are shown before, during (grey bar) and after each duration of 05s of NW_REF_ (A), 30s of NW_REF_ (B), 60s of NW_REF_ (C), 05s of SS_REF_ (D), 30s of SS_REF_ (E) and 60s of SS_REF_ (F). Responses were synchronized by the beginning of stimulation, set at 60s. For statistical analyses, shorter segments (T1-T4) were averaged from 40-50s (T1), 60-70s (T2), 110-120s (T3) and 120-130s (T4), respectively.

**Table 2:** Mean (SD) values of bilateral cerebral hemodynamic changes at each timepoint for different duration of NW_REF_ and SS_REF_ paradigms.

**CBFV**_**RH**_ **(%)**					**Variation (p-value)**		
**NW**_**REF**_ (R-word)	**T1**	**T2**	**T3**	**T4**	Interaction	Timepoints	Paradigms
05s	-0.4(1.1)	5.2(3.9)^a^	-0.6(5.8)^b^	-0.4(4.6)^b^	0.37	**<0.0001**	0.62
30s	-1.4(2.0)	6.9(4.9)^a^	1.5(7.5)^b^	-0.8(4.9)^b^			
60s	-1.3(1.7)	6.1(3.7)^a^	-2.2(5.9)^b^	-0.6(6.3)^b^			
**SS**_**REF**_ **(100–7)**	**T1**	**T2**	**T3**	**T4**	Interaction	Timepoints	Paradigms
05s	-0.6(1.8)	3.7(3.7)^a^	-3.5(3.1)^b^	-3.9(3.7)^b^	**0.002**	**<0.0001**	**0.02**
30s	-1.2(1.1)	6.4(3.7)^a^	0.0(6.2)^b^	0.4(5.6)^b^			
60s	-1.0(1.6)	4.1(4.9)^a^	3.8(6.9)^a^	3.8(9.1)^a^*			
**CBFV**_**LH**_ **(%)**					**Variation (p*-*value)**		
**NW**_**REF**_ (R-word)	**T1**	**T2**	**T3**	**T4**	Interaction	Timepoints	Paradigms
05s	-0.3(1.4)	5.8(4.8)^a^	-1.4(4.6)^b^	-1.1(3.3)^b^	0.58	**<0.0001**	0.32
30s	-0.3(0.4)	8.1(4.8)^a^	1.0(4.4)^b^	-0.2(2.5)^b^			
60s	-1.2(1.5)	6.7(2.9)^a^	0.8(7.9)^b^	0.1(6.1)^b^			
**SS**_**REF**_ **(100–7)**	**T1**	**T2**	**T3**	**T4**	Interaction	Timepoints	Paradigms
05s	-0.6(1.3)	3.8(3.7)^a^	-2.4(2.9)^b^	-3.7(5.0)^b^	**0.0057**	**<0.0001**	0.0589
30s	-1.3(1.2)	6.6(4.5)^a^	1.0(5.2)^b^	2.4(6.5)			
60s	-1.1(1.3)	4.2(3.5)^a^	3.1(6.9)^a^	2.0(8.6)			

CBFV was bilaterally normalized at baseline values. Sample size = 16, T1-T4 represents each extracted timepoint for statistical analyses. Interaction showed p-value of paradigm x timepoint effect by two-way repeated measures ANOVA followed by post-hoc analysis with Tukey’s multiple comparison. CBFV; cerebral blood flow velocity, RH; right hemisphere, LH; left hemisphere, s; second, NW_REF_; reference word-naming and SS_REF_; reference serial subtraction.

^a^ p < 0.05 for difference compared with baseline (after Tukey correction)

^b^ p < 0.05 for difference compared other timepoints with T2 (after Tukey correction)

^c^ p < 0.05 for difference between paradigm comparisons (after Tukey correction)

* p < 0.05 for difference between interhemispheric comparisons

The article "The scalability of common paradigms for assessment of cognitive function: A functional transcranial Doppler study" was published in 2022. Journal: PLoS One.

### Effect of task complexity on cerebral haemodynamic responses

Increases in the complexity of NW and SS tasks induced similar temporal CBFV changes during neural activation as no obvious difference was seen in its effect on CBFV responses within each time period of stimulation. Table 1 presents values of bilateral CBFV changes at each time segment for both NW and SS tasks, in both RH and LH. There was no significant interaction effect on bilateral CBFV responses between complexity paradigms and time segments on two-way ANOVA (Table 1). There were no significant differences between CBFV changes for NW and SS complexities at each time-point.

### Effect of task duration on cerebral haemodynamic responses

Differences in the duration of NW_REF_ and SS_REF_ tasks induced a similar pattern of temporal CBFV responses (Fig 3), with a lack of significance in its effect on CBFV changes at initial NVC activation (Table 2). Both RH and LH showed highly significant bilateral CBFV changes for both NW_REF_ and SS_REF_ (Table 2). A significant interaction was seen between timepoint and duration for the SS_REF_ in both RH (p = 0.002) and LH (p = 0.0057). As expected, due to the reduced duration of paradigms, significant differences were seen for the SS_REF_ with increasing durations in the RH (p = 0.02) at T3 and T4 and borderline significant in the LH (p = 0.059) (Table 2), but not for NW_REF_.

### Interhemispheric differences

Overall, there were contradictory responses between RH and LH regarding the dominance of CBFV responses during SS and NW tasks, respectively. Significant interhemispheric differences were observed for RH with SS and LH for NW tasks but only for the timepoints T3-T5 (Table 1). In paradigms of different complexity, CBFV response for LH was significantly greater than RH (p = 0.028) during R-words at T3. On the other hand, for SS, RH had significantly higher CBFV response than LH at T4 (100–2, p = 0.041 and 100–7, p = 0.043) and T5 (1000–17, p = 0.007). However, hemispherical differences in both NW_REF_ and SS_REF_ were not seen at each time segment during 05s and 30s durations.

## Discussion

### Main findings

As a non-invasive tool, fTCD has often been used to detect changes in cerebral haemodynamic responses during neural activation using cognitive paradigms [11, 21, 23]. In this novel study of the effects of paradigm complexity and duration, we focused on the coherent averages of CBFV, as the dominant technique that has been used for assessment of NVC with fTCD. Our main finding was that in healthy participants, the temporal CBFV response failed to demonstrate sensitivity to NW and SS cognitive paradigms of varying complexity and duration. By showing similar patterns of otherwise highly significant alterations in the CBFV response at the onset of all tasks, these changes, and the subsequent temporal evolution of the CBFV response was not consistently sensitive to detect any effect of complexity or duration with both the NW and SS paradigms. However, different CBFV responses were observed during the sustained response and at the end of stimulation, depending on the type of paradigm undertaken. More work is therefore needed to obtain a better understanding of the NVC response to these commonly used cognitive tasks and the poor sensitivity they express to changes in cognitive load.

The article "The scalability of common paradigms for assessment of cognitive function: A functional transcranial Doppler study" was published in 2022. Journal: PLoS One.

### Temporal pattern characteristics of fTCD responses to cognitive tasks

The highly significant bilateral CBFV differences observed across time (Tables 1 & 2), confirmed that these paradigms could induce NVC responses to cognitive stimulation for all subjects. The two distinct phases of the bilateral CBFV responses to paradigms of different complexity that we observed, are in agreement with the existing literature [45, 46]. Different interpretations have been given as to the mechanisms underlying the fast response observed at T2. Whilst the CBFV changes may represent effort-related cognitive processes [47], Boban *et al*. (2014) and Szirmai *et al*. (2005) proposed that fast-neurogenic regulation, with a more attention-induced arousal reaction to mental activations, resulted in the rise of perfusion pressure rather than representing a vasodilatory response to meet metabolic demand [48, 49]. However, Sato *et al*. (2001) suggested that the initial fast response at T2 resulted from direct neurogenic vasodilation resulting from free circulating acetylcholine, activation of both muscarinic and nicotinic cholinergic receptors in the cortex, and involvement of NO release from nitric oxide synthase cells such as interneurons or endothelial cells [50], which is supported by the existence of corticothalamic axons in the vascular bed of the thalamus [51]. Neurogenic regulation may therefore nourish a rapid adaptive response with uncoupling of the cortical metabolic rate during initial stimulation.

For the second peak, a gradual CBFV increase was seen as the sustained response (T3), with differences related to the complexity of NW and SS, except for SS (100–2). This slow phase of the CBFV response could reflect metabolic regulation that induced decreases in local microvascular resistance depending on the actual level of tissue CO_2_ concentration [49]. However, in SS (100–2), the absence of a second peak might be due to this being the easiest paradigm [52], combined with a desire to quickly complete the task with rapid answers and associated hyperventilation. Therefore, an attenuated CBFV response might be particularly associated with retrieving arithmetic facts in simple calculations

The article "The scalability of common paradigms for assessment of cognitive function: A functional transcranial Doppler study" was published in 2022. Journal: PLoS One.

### Influence of paradigm complexity on fTCD responses

Paradigms of different complexity induced CBFV responses with similar temporal patterns, and without significant differences in the amplitude of the CBFV changes, or evidence of lateralization (Table 1). Although our cognitive-challenging tasks did not provide CBFV responses with consistent interhemispheric differences, our findings were in line with other studies showing reduced lateralisation with increasing task difficulty, possibly due to recruitment of additional neural networks compensating for increased cognitive demands [53]. Also, most paradigms used in common cognitive assessments have not resulted in significant lateralisation [26]. On the other hand, there is evidence in the imaging literature that other techniques for NVC assessment might be more responsive to differences in cognitive effort. In fMRI investigations, the consequences of increasing complexity in verbal fluency performance showed greater activation in the anterior cingulate region [54], with activation predominantly in the right cerebellar hemisphere [55], and with laterality increased in the posterior part of the inferior frontal gyrus during mentally complex calculation [56]. This might help to explain our results with increasing complexity of NW and SS tasks, respectively. However, only the inferior frontal gyrus is part of the territory perfused by the MCA [57]. Thus, changes in CBF, resulting from paradigms of different complexity, might occur in regions other than those perfused by the MCA. As reported by Smirl *et al*. (2016), using different levels of challenge in visual search paradigms, it was possible to discriminate ΔCBFV responses in the posterior cerebral artery (PCA), but ΔCBFV changes to visual paradigms of different complexity could not be detected in the MCA [58]. Similarly, bilateral CBFV changes showed a larger response during the Stroop test with cognitive incongruent (difficult) than congruent (easy) stimuli [48]. With more demanding tasks, larger ΔCBFV was seen bilaterally during *n*-back paradigms compared to less demanding tasks [35]. Also, the differences between interhemispheric activations [49, 59, 60] could be discriminated by task difficulty. These pronounced differences probably depend on duration of stimulation, type and complexity of paradigms [26].

The article "The scalability of common paradigms for assessment of cognitive function: A functional transcranial Doppler study" was published in 2022. Journal: PLoS One.

Noteworthy, the majority of previous studies used repeated presentations of the same paradigm to improve signal-to-noise ratio (SNR) of intra-subject averages of the ΔCBFV response. As seen in previous studies, presentation of complex tasks was repeated a variable number of times, including < 5 [59], 5 to 10 [24, 48, 49, 54–56, 61, 62] or > 10 times [60]. Studies with repeated task presentation were likely to provide more consistent responses across individuals, as compared to the present study where tasks were presented only once.

There are potential additional explanations for the lack of significance in our results to the effects of cognitive load with NW and SS paradigms. First, the differences in complexity of paradigms in the current study might not have been sufficient to induce differential CBFV responses, as proposed in terms of the *compensation-related utilization of neural circuits hypothesis* (CRUNCH) to recruit more neural activations matching with load increases [63, 64]. As reported for other neuroimaging techniques (fMRI or SPECT), it provided greater activation in some specific brain areas, with increased task difficulty with verbal [54], arithmetic [56] or visual [30, 65] paradigms. Although NVC assessment with fTCD has been rated as equivalent to that obtained with fMRI [66], this does not seem to be the case in our study, with respect to the ability of fTCD to reflect differences in complexity. We can speculate that increasing tasks difficulty cannot induce the CRUNCH effect on TCD-measured CBFV changes.

Secondly, the phenomenon of ‘central command’ anticipation of the brain when preparing to receive an increased demand for oxygen may be important. To our knowledge, the role of the ‘central command’ during cognitive paradigms in fTCD studies has received very little attention in the human NVC literature [67]. Previous studies suggested that the preparatory process of blood flow adjustment involves alertness of attentional function [68], correlated with increasing CBF response before the onset of exercise that is likely governed by the ‘central command’ network [69]. Therefore, increased CBFV at the onset of all paradigms, independently of complexity or duration, was probably determined by the effects of ‘central command’ on the neurovascular unit.

Thirdly, cognitive stimulation of some brain areas leads to inhibition of other cortical centres [70]. Despite the cerebral cortex circulation supporting the local metabolism during cognitive activation [71], there is evidence in the literature showing a decreased activation in the medial prefrontal, precuneus, posterior cingulate and left angular gyrus, near to Wernicke’s area (language function), following increased cognitive load of NW tasks [72]. Similarly, Menon *et al*. (2010) highlighted a shift in the process of brain response from prefrontal cortex to the bilateral posterior parietal cortices, including additional brain areas (caudate nucleus and cerebellum) during complex mental arithmetic [73]. It is plausible that the impact of increasing cognitive complexity might be a true decrease in some local brain areas [72, 73]. The expected increased response in CBFV following stimulation might therefore be overshadowed by the increase in inhibition with greater cognitive demand. Finally, increases in the amplitude of the CBFV response, following cognitive paradigms of increasing complexity, could have been confounded by concomitant changes in systemic covariates. The influence of sympathetic activation inducing a rise of BP and HR during cognitive paradigms has previously been reported, and changes in EtCO_2_ with hypocapnia-induced hyperventilation or hypercapnia-induced breath holding can also accompany CBFV alterations during cognitive tasks [21, 74]. Furthermore, increases in HR were reported at the beginning of more complex cognitive tasks [48], resulting from arousal or stress. The contribution of BP and PaCO_2_ to CBFV changes following cognitive tasks has been confirmed in previous fTCD studies [75]. However, whether these co-variates can obscure the changes in CBFV response that could be expected with increasing complexity needs to be investigated with the use of more advanced multivariate dynamic modelling techniques.

The article "The scalability of common paradigms for assessment of cognitive function: A functional transcranial Doppler study" was published in 2022. Journal: PLoS One.

### Influence of paradigm duration on fTCD responses

For our hypothesis regarding paradigms of different durations, it would be expected that shorter or extended duration paradigms would result in different magnitude changes of CBFV following cognitive activation. With different durations for both NW_REF_ and SS_REF_, temporal CBFV responses showed similar patterns at the first peak of initial stimulation (T2), without significant differences in the amplitude of CBFV or lateralized dominance. Only CBFV responses to the longer (60s) stimulations led to a second peak for SS_REF_ (Table 2). Despite the 60s stimulation being more likely to induce greater metabolic demand, than 5s and 30s durations, the magnitude of CBFV changes was lower than for stimulation with 30s duration (Fig 3). These results were consistent with previous studies of different durations of stimulation, which demonstrated that the longer duration stimulation would not necessarily maximize the CBFV magnitude change [29, 76].

To our knowledge, there have been no previous fTCD studies of the effects of changing cognitive paradigm duration on the induced changes in CBFV. However there have been previous TCD studies using visual stimulation of different durations [62, 76, 77]. The results of these studies were consistent, showing an identical curve of CBFV response at the initial phase, independent of the duration of stimulation, as seen in other imaging literature (e.g. BOLD) [10, 78, 79] and our paradigms. According to the ‘central command’ hypothesis, the lack of marked differences in CBFV responses with varying durations could be explained by the anticipatory response to cognitive demand in the attentional process [68], governing an upsurge of CBFV around 5s after onset stimulation, without further influence of the duration of stimulation on the NVC mechanism.

In tasks with 60s duration, a slow CBFV peak was found in both hemispheres before T3 in SS_REF_ (Fig 3). This is in contrast to CBFV patterns seen in previous studies with stimuli of varying duration, that demonstrated a plateau phase with longer duration stimulation, using both fTCD [62] and BOLD [79]. The difference in CBFV responses might depend on the type of paradigm. The plateau curve might relate to an adaptative brain response as a compensatory function [80, 81], but the two-peaked pattern in CBFV response seen in our and other studies [46, 48] might be confounded from involuntary hyperventilation-induced hypocapnia after the first peak [45, 48, 82] which affects approximately 30s of the magnitude of the CBFV response. Accordingly, a second peak will be missing in paradigms of shorter (5s and 30s) duration.

### Clinical implications and limitations

This is the first systematic study to determine fTCD-measured NVC responses to NW and SS paradigms of varying complexity (easy, moderate and hard) and duration (shorter, intermediate and longer) by modifying well known paradigms used for clinical assessment of cognitive performance [37–39, 41]. The results suggest that fTCD, based on a single presentation of a paradigm, provides questionable results, regarding its feasibility to detect alterations in mild cognitive impairment (MCI) and other conditions. From previous studies in our group, Beishon *et al*. (2018) demonstrated a significant decrease of CBFV at sustained response during a language task in Alzheimer’s disease but not in MCI when compared with healthy controls [19]. Although the mean of repeated task presentations to each patient might provide more robust estimates of the CBFV changes [83, 84], combining the use of fTCD with other modalities (EEG or near infrared spectroscopy) may enhance discriminatory power in clinical NVC studies [85]. These and other alternatives need to be explored further to provide greater confidence in the use of fTCD in clinical studies of NVC.

The article "The scalability of common paradigms for assessment of cognitive function: A functional transcranial Doppler study" was published in 2022. Journal: PLoS One.

There are a number of limitations to our study. First, TCD reflecting CBFV changes in the MCA, can be directly proportional to changes in absolute CBF with the assumption that the diameter of insonated MCA remains constant despite small changes in CO_2_ and BP [86, 87]. Second, fTCD measurements limited to the MCA might not have the same sensitivity to cognitive stimulation as techniques with greater spatial resolution, such as PET or fMRI [21]. One interesting possibility would be to perform simultaneous measurements in the MCA and PCA as an attempt to improve sensitivity. Third, language task difficulty has been reported to have reduced sensitivity [88, 89], although Payne *et al*. (2015) showed differences in fTCD responses to the joint fast paced presentation of rhyme and line array judgement tasks [90]. It is possible that the level of difficulty used in our NW paradigms was insufficient to induce differential changes in CBFV responses in the MCA. In addition, the motivation level of participants to engage and perform the tasks to the best of their ability could have affected their CBFV responses, despite our encouragement prior to each test. The role of personal motivation, and how it could be individually assessed, is complex and warrants further investigation [91]. Fourth, the education level could be an important co-variate of cognitive performance. We have not taken this aspect into consideration, given the homogeneity of educational background in our sample, with all participants having had between 16 and 22 years of education. A recent review has highlighted inconsistent findings in previous studies about the effect of ageing on cognitive function [5]. For this reason, further studies are needed to understand the influence of ageing in healthy older adults, and its interaction with the NVC response to tasks with varying complexities and durations. Finally, another limitation was the relatively small sample size (n = 16). However, previous sample size calculations showed that 14 participants could detect a difference of 2% in CBFV at 80% power with p = 0.05, for the case of the P-words task of 60s duration [26]. Although our sample size was approximately the same, it is possible that much larger numbers are needed to detect the subtle differences resulting from NW tasks of greater or lesser complexity in comparison with naming P-words.

The article "The scalability of common paradigms for assessment of cognitive function: A functional transcranial Doppler study" was published in 2022. Journal: PLoS One.

## Conclusions

We have demonstrated that complexity and duration of NW and SS paradigms provided similar patterns and amplitudes of CBFV responses, without the possibility of making a scalable metric for assessment of NVC in healthy subjects. Nevertheless, some significant changes were seen in comparison with SS_REF_ for the effects of different task durations, indicating a complex interaction between NVC response and duration of stimulation. Further studies, on the sensitivity of the fTCD response to stimulation of varying complexity and duration, is needed by performing similar studies in the influence of ageing, patients with early signs of MCI, Alzheimer’s disease or other types of dementia, exploring alternative cognitive paradigms. Also, a more integrated approach as described previously [22, 24, 92] is needed to take into consideration the potential contribution of other determinants of CBFV, such as BP and EtCO_2_, to identify parameters of the NVC response that could be scalable, ideally in a linear fashion.
